# Acrid and Bitter Chinese Herbs in Decoction Effectively Relieve Lung Inflammation and Regulation of TRPV1/TAS2R14 Channels in a Rat Asthmatic Model

**DOI:** 10.1155/2022/8061740

**Published:** 2022-08-22

**Authors:** Yamei Yuan, Xiangming Fang, Weidong Ye

**Affiliations:** ^1^Graduate School, Anhui University of Traditional Chinese Medicine, Hefei, Anhui, China; ^2^Clinical College of Traditional Chinese Medicine, Anhui University of Traditional Chinese Medicine, Hefei, Anhui, China

## Abstract

**Background:**

Shegan Mahuang decoction (SGMHD) was widely used as a classic prescription of traditional Chinese medicine to treat asthma. However, there is no research on the acrid and bitter Chinese herbs in the SGMHD to treat asthma. This study aimed to investigate the effects of SGMHD and its acrid-bitter Chinese herbs composition on airway inflammation and the expression of TRPV1 and TAS2R14 genes and proteins in asthmatic rats.

**Methods:**

SD (Sprague Dawley) rats of asthma were induced by ovalbumin and aluminum hydroxide, then randomly divided into the Normal group, Model group, SGMHD group, Dexamethasone (Dex) group, Guilongkechuangning (GLKC) group, The Acrid Chinese Herbs group (ACH), and The Bitter Chinese Herbs group (BCH). The rats were given intragastric gavage after 21 days for 4 weeks. The bronchoalveolar lavage fluid (BALF) was collected, and the levels of IL-4, IL-13, nerve factors SP, CGRP, PGE2, and serum of IgE were determined by ELISA. Pathological changes in the lungs were determined by hematoxylin-eosin (HE) staining. The expression of TRPV1 and TAS2R14 in the rat lung group was detected by immunofluorescence (IF). The expression levels of TRPV1 and TAS2R14 were measured using western blotting. The mRNA levels of TRPV1 and TAS2R14 were measured using RT-qPCR.

**Results:**

The levels of serum IgE in treated rats and the cytokines IL-4, IL-13, SP, CGRP, and PGE2 were all decreased. HE-staining showed that significantly reduced inflammatory cell infiltration in lung tissue. IF-staining showed the expression levels except those of the normal group were enhanced. Acrid Chinese herbs inhibited TRPV1, and bitter Chinese herbs activated the gene and protein expression of TAS2R in the lung.

**Conclusion:**

The acrid Chinese herbs regulate TRPV1, and bitter Chinese herbs regulate the gene and protein expression of TAS2R14, through nerve and immune-inflammatory factors, reduced airway inflammation, reduced airway reactivity, promoted airway remodeling, and the combination of acrid-bitter Chinese herbs can enhance the above effects. This will lay a foundation for further in vivo study of specific compounds of acrid-bitter Chinese herbs.

## 1. Introduction

Asthma is characterized by airway hyperresponsiveness caused by various stimuli, airway inflammation, and airway structural changes caused by reversible airway constriction [1]. According to the survey, the prevalence of asthma worldwide is increasing and epidemic year by year [2]. In the 25 years prior to now, there was a significant increase in asthma incidence by +19.8% and asthma prevalence by +28.8% [3]. SGMHD was Zhang Zhongjing's prescription in the Han Dynasty, which contains nine traditional Chinese herbs (*Ephedra sinica* Stapf, *Asarum sieboldii* Miq., *Pinellia ternata* (Thunb.) Breit., *Tussilago farfara* L., *Zingiber officinale* Roscoe., *Aster tataricus* L.f., *Belamcanda chinensis*, *Ziziphus jujuba* Mill, and *Schisandra chinensis* (Turcz.) Baill. (L.) Redouté) [4], including acrid and bitter ones. It was widely used in the treatment of a variety of respiratory diseases and has a certain clinical effect. The components of SGMHD's preliminary studies showed that HPLC fingerprints which have 22 peaks recorded contained guanosine, chlorogenic acid, tectoridin, 6-gingerol, and Wuweizisu B [4]. However, there are few clear reports about the effect and mechanism of its component group of acrid-bitter Chinese herbs taste on asthmatic rats [5].

TRPcation channel subfamily V member 1(TRPV1) is a ligand-gated nonselective cationic channel that can be activated by various exogenous and endogenic physical and chemical stimuli, both in bronchial epithelial cells and lung tissues [6]. In current animal models and patients with asthma, its expression has been found to be elevated, and its inhibitors can alleviate airway inflammation [7]. The TRPV1 ion channel is the hub of almost all neuronal inflammatory signaling pathways, and there is evidence that there is two-way feedback between immunogenic and neurogenic mechanisms in airway inflammation, including subsubstance P (SP) and calcitonin gene-related peptide (CGRP) [8]. Because of its ability to be activated and functionally sensitized by proinflammatory mediators and harmful stimuli, TRPVI is considered to be a pathological receptor that plays an important role in the transduction of harmful stimuli and the maintenance of inflammatory states [9]. At the present stage, studies have found that TRPV1 can be activated by capsaicin in acrid traditional Chinese herbs pepper and Evodia rutaecarpa in Evodia rutaecarpa alkalies, such as gingerol diol compounds, 2-nonanone, and paradol, all of which come from ginger [8]. Among the active ingredients targeted by the pharmacophore model of TRPV1 agonist, 60.11% belonged to the acrid Chinese herbs, which indicated that the pharmacophore model could characterize the common structural characteristics of acrid Chinese herbs components to a certain extent, and had a certain ability to distinguish acrid Chinese herbs components [10, 11].

Recent studies have shown that there are bitter taste receptors (TAS2Rs) on human airway smooth muscle (ASM), lung, and ciliated epithelial cells [12–14]. TAS2R mediates the production of bitter taste in taste buds [15, 16]. Previous studies have reported that TAS2R14, the first receptor identified to exhibit a broad beta 2(*β*2) agonist spectrum, has the highest expression level in human bronchi among the 25 TAS2Rs [17]. The use of TAS2R agonist can inhibit the secretion of cytokines by immune cells and reduce airway inflammation [18–20]. TAS2R14 agonists have been reported to induce significant effects on airway smooth muscle relaxation [17, 21, 22], and direct TAS2R14 agonists can inhibit IgE-dependent mast cell activation [22, 23], Therefore, the microcosmic and molecular mechanism of the effect of bitter Chinese herbs may be correlated with TAS2Rs to some extent [24].

At present, glucocorticoids and *β*2 receptor agonists are mainly used in the treatment of asthma, but long-term use will cause adverse reactions [25], and about 40 percent of asthma patients do not respond to corticosteroids [26–28]. SGMHD, a classic prescription, has been used to relieve asthma symptoms for about 2,000 years [29–31]. The study revealed that SGMHD may treat asthma by regulating the production of inflammatory mediators [32]. Therefore, this study provides a new understanding of the mechanism by which SGMHD and its acrid-bitter Chinese herbs component regulate antiairway inflammation through TRPV1/TAS2R14.

## 2. Materials and Methods

### 2.1. Drugs and Reagents

The components of SGMHD include nine herbs, acrid Chinese herbs (*Ephedra sinica* Stapf, *Asarum sieboldii* Miq., *Pinellia ternata* (Thunb.) Breit., *Tussilago farfara* L., and *Zingiber officinale* Roscoe) and bitter Chinese herbs (*Aster tataricus* L.f. and *Belamcanda chinensis*) [4]. In this experiment, the SGMHD, the acrid herbs group, and the bitter herbs group were made by the First Affiliated Hospital of the Anhui University of Chinese Medicine. GuiLongKeChuangNing (GLKC) (specification, 0.41 g/tablet) (Ren He Pharmaceutical Co., Ltd., Jiangxi, China), dexamethasone (Dex) (specification, 0.75 mg/tablet) (South Land Pharmaceutical Co., Ltd., Guangdong, China), ovalalbumin (OVA) (No. A5253, Sigma's Louis, MO, USA), and aluminum hydroxide (No. 2001060, Sinopharm Chemical Reagent, Hebei, China).

### 2.2. Animals

70 male Sprague Dawley (SD) rats (150–180 g) were purchased from the Hangzhou medical college (Hangzhou, Zhejiang, China), with certification No. SCXK (Zhe) 2019-0002. The rats were acclimated to the conditions (temp: 22–24°C, relative humidity: 50%–70%) for one week before experiments commenced, and then randomly divided into the Normal group, Model group, SGMH group (which contains the acrid Chinese herbs and the bitter Chinese herbs), Dexamethasone group (Dex) , GLKC (GuiLongKeChuangNing) group, the Acrid Chinese Herbs group (ACH), and the Bitter Chinese Herbs group (BCH). Each group contained 10 rats. All animal procedures were approved by the Ethical Committee for the Experimental Use of Animals at the Anhui University of Chinese Medicine (Hefei, Anhui, China, approval AHUCM-rats-2021058).

### 2.3. Establishment of Rat Allergic Asthmatic Model

The rat model of allergic asthma was induced by ovalbumin sensitization in this study. On days 1 and 14, rats were sensitized by intraperitoneal injection of 1 ml antigen sensitization liquid containing 10% OVA diluted in sterile normal saline and 10 mg aluminum hydroxide as an adjuvant, respectively, in the abdominal cavity and both sides of the inguinal subcutaneous. On the 15th day, rats inhaled 1% OVA for 30 minutes once daily and were intermittently placed in an adjustable cold chamber (0–2°C) After the end of the atomization, the rats showed obvious nodular wheezing, abdominal muscle convulsions, and even unstable standing, which indicated an acute asthma attack, for consecutive 3 weeks, while rats in normal and model groups were given an equal volume of NS.

### 2.4. Administration of Drugs and Sample Collection

From the 36th day of modeling, the normal and asthma group were intragastrically administrated with 10 ml/kg/d normal saline (NS), while rats in the experimental groups were administrated with 6.43 g/kg/d SGMHD, acrid Chinese herbs and bitter Chinese herbs, 10 g/kg/d GLKC tablets as well as 0.5 mg/kg/d Dex per day for 21 successive days. The rats were fasted for 24 h, inhaled OVA, and anesthetized with 2% pentobarbital (20 mg/100 g) (Shanghai Chemical reagent procurement and supply station, 20210516). Blood, lung tissue, and BALF (bronchoalveolar lavage fluid) were collected for further study.

### 2.5. Measurement of Cytokines in BALF and Serum IgE Levels

IgE (JYM0441Ra) in serum, IL-4 (JYM0647Ra), IL-13 (JYM0477Ra), SP (JYM0328Ra), CGRP (JYM0375Ra), and PGE2 (JYM0446Ra) in BALF were detected by enzyme-linked immunosorbent assay (ELISA, Wuhan ColorfulGene Biological Technology Co., Ltd., Wuhan, China). The collected blood (5ml) and balf (1000g) were allowed to stand at temperature for 2 h and centrifuged for 15 min (4°C). The serum was diluted according to the kit instructions, and the BALF supernatant was dissolved on ice and then diluted. Then, the reaction system was added. Finally, the concentrations of IgE in the serum were calculated, and the levels of inflammatory cytokines in balf were analyzed in each group.

### 2.6. Hematoxylin-Eosin (HE) Staining

Lung tissues were fixed in 4% formaldehyde, cut into 5 *μ*m sections, and stained with hematoxylin and eosin (HE), then to observe the morphological changes in lung tissues and inflammatory cell infiltration under an optical microscope (Olympus Optical Co., Ltd., Tokyo, Japan).

### 2.7. Immunofluorescence Staining

The slices were baked for 20–30 min, then 3 lines of xylene (5 min) were added, and three lines (100%–95%–80%) of ethanol (3 min) were administered successively. After washing, the antigen was repaired under high pressure. After washing 3 times with PBS T, 0.5% TritonX-100 (Ebiogo, 06282118) was dropped and incubated for 30–60 min at 37°C. Goat serum was sealed, and primary antibody TRPV1 (Bioworld, BS60454) and TAS2R14 (Bioss, ab138271) were dropped for 60 min at 37°C. PBS T was rinsed, and a secondary antibody (goat anti-rabbit IgG (FITC)/1: 400) (Ebiogo, 06292105) was dropped for 30 min at 37°C. The slices were sealed piece with an anti-fluorescence quenched blocking agent (including DAPI). A digital slice scanner (Pannoramic MIDI) scanned fluorescent slices.

### 2.8. Western Blot Analysis

Total protein samples were extracted from lung tissue cells using RIPA lysis buffer. Concentrated glue, separation glue, carding, sample loading, electrophoresis, film transfer, quantitative detection were prepared by the BCA method, adding different primary antibody and secondary antibody, respectively (diluted strictly according to the instructions), closed at room temperature for 2 h, adding PBST detergent. Rats TRPV1 (1 : 1000, Bioworld, USA), TAS2R (1 : 1000, Abcam, UK), and GAPDH (1 : 1000, Zeb-io, China) antibodies were added for incubation overnight and washed 3 times, 10 min for each washing. After ECL color development, the film was exposed and analyzed with Image J software. The experiment was repeated 3 times [33]. The protein levels of TRPV1 and TAS2R were detected.

### 2.9. Reverse Transcription-Quantitative PCR Analysis

Lung tissue (50 mg) was cut into fragments and placed in a centrifuge tube. Total RNA was extracted with Trizol (Life Technologies, Carlsbad, CA, USA) reagent, and its integrity was detected by electrophoresis. The instructions of the PrimeScript™ RT reagent kit with gDNA Eraser were followed (Takara Bio Inc., Shiga, Japan), transcribing cDNA, amplifying, and synthesizing the target fragment with DNA polymerase. The amplification conditions were denatured at 95°C for 10 min and 95°C for 20 s, 40 cycles, then annealed at 60°C for 1 min. After the reaction, the data were analyzed, and the mRNA expression level was calculated by using the 2−ΔΔ CT method [34]. GAPDH was taken as an internal reference. The primer sequence was as follows:

  TRPV1-F, 5′-GCAAGAAGCGCCTGACTGAC-3′
  TRPV1-R, 5′-CAGGAGCAGAGCGATGGTGT-3′
  TAS2R14-F, 5′-CTTTGGCCCTTACCAGACTC-3′
  TAS2R14-R, 5′-ACCCAGATAACACCTATCGC-3′

### 2.10. Technical Roadmap of Experimental Research on Asthma Intervention by SGMHD

The technology roadmap is shown in Figure 1. On days 0, 7, and 14, the rats were sensitized by injecting 10% OVA intraperitoneally and subcutaneously in the bilateral groin, respectively, and the animal models were established. On the 15th day, inhalation and nebulization of 1% OVA were started. After 21 days of modeling, rats were randomly selected for HE-staining, which confirmed the success of the model. Then, the intragastric treatment was performed for 3 weeks. BALF, serum, and lung tissue were collected for subsequent experimental studies. No rats died during the modeling process.

### 2.11. Statistical Analysis

The data were analyzed using SPSS 22.0 software (SPSS, Inc., USA) and Graphpad 8.0 which are shown as (mean ± standard) deviation. Differences between 2 groups were compared by two-tailed *t*-test, and ANOVA and Tukey tests were used to determine the differences between groups. *P* < 0.05 was considered to be a statistically significant difference.

## 3. Results

### 3.1. General Information about Animals

The Normal group rats had a normal diet and all activities, while the model group rats had symptoms such as restlessness, hair erect, rapid breathing, cyanosis, abdominal spasm, and limp limbs. In the other groups, compared with the model group, the above symptoms were not obvious, and the general activities such as mental ability, diet, and water intake were normal.

### 3.2. ACH and BCH Alleviate Airway Inflammation in Asthmatic Rats

Compared with the Normal group (Figure 2), the pathological changes of lung tissues in the model group (Figure 2) were obvious, including a large number of inflammatory cell infiltration, lung bullae atrophy or disappearance, incomplete alveolar structure, and substantial changes in some lung tissues, but compared with the Model group, the above histopathological changes were significantly improved in SGMH group, Dex group, GLKC group, ACH group, and BCH group (Figures 2(c)–2(g)). Through IF staining, compared with Normal group TRPV1, the expression of ACH and BCH was increased in the Model group, but decreased significantly in the SGMH group (*P* < 0.001, *P* < 0.05). Compared with the Normal group's TAS2R14, the expression of ACH and BCH was decreased in the Model group and increased in the SGMH group (Figure 3), and the positive expression positions were red.

### 3.3. ACH and BCH Downregulate the Expression of Immune- and Neuro-Related Factors

Elevated levels of inflammatory cytokines are characteristic of airway pathology in asthma. Therefore, to evaluate the efficacy of SGMHD and acrid, bitter Chinese herbs in treating asthma inflammation in rats, the IgE in serum and IL-4, IL-13, SP, CGRP, and PGE2 levels in BALF were detected with an ELISA kit. From the data, the treatment of SGMH (ACH + BCH), ACH, or BCH reversed the increased IgE (*P* < 0.001), IL-4 (*P* < 0.001), IL‐13 (*P* < 0.001), SP (*P* < 0.001), PGE2 (*P* < 0.001), CGRP (*P* < 0.001) levels (Figures 4(a)–4(f)). Among them, compared with the SGMH group, there were significant differences in IgE, IL-4, IL-13, SP, PGE2, and CGRP in the ACH group (Figures 4(a)–4(f)) (*P* < 0.001, *P* < 0.05), IL-4 had a statistical difference in the BCH group (Figure 4(b)) (*P* < 0.001). Compared with the GLKC group, IL‐4 was statistically different in the SGMH group (*P* < 0.001) (Figure 4(b)), IgE, IL-4, IL‐13, and CGRP were significantly different in the ACH group (*P* < 0.001, *P* < 0.05) (Figures 4(a)–4(f)). Compared with the Dex group, IL‐4 was significantly different in the SGMH group (*P* < 0.001) (Figure 4(b)). IgE, IL‐13, SP, and CGRP were significantly different in the ACH group (*P* < 0.001, *P* < 0.05) (Figures 4(a)–4(d) and 4(f)). In conclusion, ACH and BCH can reduce inflammatory factors, and the combined use of ACH and BCH has a better effect.

### 3.4. Acrid-Bitter Chinese Herbs Regulate TRPV1/TAS2R14 in Lung Tissue of Rats

The gene expression of mRNA in lung tissues was detected by the RT-qPCR, and the 2-ΔΔCT method was used to analyze the data. Compared with the Normal group, the expression of TRPV1mRNA significantly increased in the model group (*P* < 0.001,*P* < 0.05) (Figure 5(a)), while TAS2R14mRNA decreased clearly (*P* < 0.001) (Figure 5(b)). After treatment, compared with SGMH, TRPV1 and TAS2R14 were statistically different in ACH and BCH groups (*P* < 0.001, *P* < 0.05) (Figures 5(a) and 5(b)). Compared with the GLKC group, TRPV1 of ACH and BCH groups showed statistical difference (*P* < 0.001) (Figure 5(a)), and TAS2R14 in the ACH group had a statistical difference (*P* < 0.001) (Figure 5(b)). Compared with the Dex group, TRPV1 in ACH and BCH groups showed statistical difference (*P* < 0.001) (Figure 5(a)), and TAS2R14 in the BCH group was statistically different (*P* < 0.001) (Figure 5(b)). In the Model group, the expression of TRPV1 protein was significantly increased (*P* < 0.001, *P* < 0.05) (Figure 6(a)), while TAS2R14 was more reduced than that in the Normal group (*P* < 0.001) (Figure 6(b)). After treatment, the expression of TRPV1 protein decreased, and the protein expression of TAS2R14 increased in each treatment group (*P* < 0.001). Compared with the SGMH group, TRPV1 was statistically different in the ACH group (*P* < 0.05) (Figure 6(a)), and TAS2R14 was statistically different in ACH and BCH groups (*P* < 0.001, *P* < 0.05) (Figure 6(b)). Compared with GLKC and Dex groups, TAS2R14 in the ACH group was statistically different (*P* < 0.001) (Figure 5(b)). In addition, the combination of ACH and BCH (SGMH group) was more effective than the other treatment groups (*P* < 0.001) (Figures 5 and 6).

## 4. Discussion

Traditional Chinese medicine (TCM) has been shown to have a therapeutic effect on asthma [31]. SGMHD was widely used in the treatment of a variety of respiratory diseases, and has a certain clinical effect; however, there are few clear reports about the effect and mechanism of its component group of acrid-bitter Chinese herbs on asthmatic rats [32]. Previous studies have found that the active components of acrid Chinese herbs can be recognized by TRPV1 and TAS2R is the main receptor that mediates bitter Chinese herbs. Meanwhile, most Chinese medicines used to treat asthma have characteristics of a bitter taste. Therefore, the TRPV1 ion channel is considered to be a potential target for the effect of acrid herbs. For asthma patients, it is necessary to find a bitter substance that can be used.

TRPV1 plays an important role in the development of asthma. Irritant gases such as vanillic acid analogies can trigger subsequent inflammatory pathways by activating TRPV1, leading to asthma [35, 36]. When TRPV1 is activated by the stimulation signal, its central hole conformation changes, causing Ca^2+^ influx, resulting in increased intracellular Ca^2+^ concentration, and integrating the upstream stimulation signal into intracellular Ca^2+^ signal, mediating the downstream nerve and immune response through neurogenic inflammation and immunogenic inflammation, inducing a series of asthma symptoms [37]. Various neuropeptides released by neurogenic inflammation have different stimulative effects on asthma. The effect of SP can increase the permeability of airway microvessels and promote the exudation of plasma protein and inflammatory cells. SP also has a strong stimulative effect on airway mucosa, leading to excessive secretion of airway mucus [38]. CGRP causes airway congestion and edema by activating the CGRP receptors in the airway vessels.

Among the five flavors of Chinese medicine, there are a large number of acrid Chinese herbs widely used in clinical practice. There is a matching relationship between the pharmacodynamic components of acrid Chinese herbs and the pharmacodynamic group model of TRPV1 agonist; the acrid Chinese herbs group is an important part of SGMHD. Mori et al. [39] found that in the asthma model, the number of IgE and Th2-related cytokines in the TRPV1 knockout group were significantly higher. This suggests that TRPV1 attenuates the Th2 immune response and inhibits the development of allergic airway inflammation, possibly because somatostatin and CGRP play a role in limiting inflammation and immune response [40]. The results of this study confirmed that SGMHD and its acrid Chinese herb can reduce airway reactivity, reduce pathological damage to lung tissue, reduce inflammatory cell infiltration, reduce Th2-related IL-4 and IL-13 cytokines levels in BALF, and regulate TRPV1 and TRPV1mRNA and protein expressions in lung tissue of asthmatic model rats, and CGRP and SP levels. It can also inhibit IgE synthesis and regulate the role of excessive immune response.

TAS2R is a G protein-coupled receptor, and different bitter substances can bind to TAS2R to cause the same bitter taste. Bitter receptors on the smooth muscle of the human airway can sense bitter substances to dilate the bronchi in the lungs and relax airway smooth muscle more efficiently than *β*2 receptor agonist [41]. Recent studies have shown that limonin can increase the expression of TAS2R14 and inhibit the production and release of related cytokines in trachea and lung tissues of rats with chronic airway inflammation caused by PM2.5 [42, 43]. These results indicate that the bitter components of traditional Chinese medicine can induce the activation of bitter receptors in respiratory tissues and inhibit the production and release of inflammatory factors, suggesting that they may be involved in the anti-inflammatory process of bitter substances [44]. It has recently been discovered in airway epithelium and smooth muscle cells [45]. Bitter agonist-induced airway relaxation has been documented in animal studies [46, 47], and research with human airway tissues also showed concordant results [44, 48–50].

Previous studies have shown that TAS2R increase in TAS2R agonists reduces the production of these inflammatory factors in a dose-dependent manner [51], and activating TAS2R inhibits airway inflammation in asthma [52, 53]. Repeated inflammatory damage and tissue repair can lead to airway remodeling, and TAS2R inhibits certain inflammatory factors [53]. The results of this study confirmed that SGMHD and its bitter Chinese herbs can reduce Th2-related IL-4 and IL-13 cytokines in BALF by regulating TAS2R14, TAS2R14mRNA, and protein expressions in lung tissues of asthmatic model rats. Inhibition of IgE synthesis and regulation of excessive immune response, regulation of CGRP and SP levels, thereby reducing airway reactivity, inflammatory cell infiltration, and lung tissue damage. So, the transcription inhibition of bitter taste receptors and its downstream signal transduction molecules is related to the occurrence of asthmatic diseases, activating the suppressed bitter taste signal transductive system may reduce inflammation, reduce respiratory mucin secretion, and prevent respiratory tissue lesions through immune-neuroregulation, so as to reduce or ease the occurrence of asthmatic diseases. In this study, the mechanisms of ACH, BCH, and their combination (SGMHD) on asthma inflammation and regulation of TRPV1 and TAS2R14 were discussed from the level of animal experiments. There is still a lack of material-based studies on the specific effects of different drug components.

## 5. Conclusion

In this study, the acrid Chinese herbs (ACH) exert an inhibitory effect on TRPV1 channels to reduce the secretion of inflammatory and alleviate airway inflammation, while bitter Chinese herbs (BCH) through regulated and inhibited the secretion of cytokines by immune cells through TAS2R, thus alleviating airway inflammation (Figure 7). The combination of SGMHD (ACH + BCH) can achieve better results, and was shown to improve asthma symptoms. In the later stage, the main components of ACH and BCH will be studied from the level of cells, how to regulate TRPV1 and TAS2R14 to improve calcium homeostasis, and regulation to improve the asthma rat model was further verified.

## Figures and Tables

**Figure 1:** The workflow of this study.

**Figure 2:** Histopathological changes in rats' lung (HE-staining, ×400, ×200). (a) In rats in the normal group, there was no abnormality in the structure of the bronchus and alveoli. (b) In the asthma rats sensitized with OVA, the bronchus was significantly thickened, and there was severe inflammatory cell infiltration in the blood vessels and peribronchial areas. Severe pulmonary inflammation and mucous production were notably reduced in rats treated with SGMH (ACH + BCH), ACH, BCH, dexamethasone (Dex), and GLKC (c–g).

**Figure 3:** Immunofluorescence changes in rats' lungs (IF-staining, ×200). Compared with the Normal group (normal), the protein expression levels of TRPV1 (a–g) and TAS2R14 (a–g) in lung tissues of rats in other groups were increased, and the nuclei were blue and the positive expression sites were red.

**Figure 4:** The level of serum IgE (a) and the level of IL-4, IL-13, SP, PGE2, and CGRP in BALF (b–f). The NS group was the negative control (normal), and the Model group (model) was the control group; SGMHD, Shegan Mahuang decoction; ACH, the acrid Chinese herbs group; BCH, the bitter Chinese herbs group represented experimental groups, and the Dex (dexamethasone) and GLKC (guilongkechuanning) groups served as the positive control groups. ^*∗*^*P* < 0.001, ^*∗∗*^*P* < 0.05 (vs normal group), ^#^*P* < 0.001, ^##^*P* < 0.05 (vs model group), ^Δ^*P* < 0.001, ^ΔΔ^*P* < 0.05 (vs SGMH group), ^a^*P* < 0.001, ^b^*P* < 0.05 (vs GLKC group), ^c^*P* < 0.001, ^d^*P* < 0.05 (vs dex group).

**Figure 5:** (a, b) The TRPV1 and TAS2R14 mRNA expressions of each group were analyzed by RT-qPCR. SGMHD, Shegan Mahuang decoction; ACH, the acrid Chinese herbs group; and BCH, the bitter Chinese herbs group, were represented as experimental groups, and the Dex (dexamethasone) and GLKC (guilong kechuanning) groups served as the positive control groups. ^*∗*^*P* < 0.001, ^*∗∗*^*P* < 0.05 (vs normal group), ^#^*P* < 0.001, ^##^*P* < 0.05 (vs model group), ^Δ^*P* < 0.001, ^ΔΔ^*P* < 0.05 (vs SGMH group), ^a^*P* < 0.001 (vs GLKC group), ^c^*P* < 0.001 (vs dex group).

**Figure 6:** (a, b) The TRPV1 and TAS2R14 protein expressions of each group were analyzed by western blot. GAPDH was used as the internal reference control. (c) The gray value of TRPV1, TAS2R14, and protein expressions was quantified. SGMHD, Shegan Mahuang decoction; ACH, the acrid Chinese herbs; and BCH, bitter Chinese herbs groups were represented as experimental groups, and the dex (dexamethasone) and GLKC (guilongkechuanning) groups served as the positive control groups. ^*∗*^*P* < 0.001, ^*∗∗*^*P* < 0.05 (vs normal group), ^#^*P* < 0.001, ^##^*P* < 0.05 (vs model group), ^Δ^*P* < 0.001, ^ΔΔ^*P* < 0.05 (vs SGMH group), ^a^*P* < 0.001, ^b^*P* < 0.05 (vs GLKC group), ^c^*P* < 0.001, ^d^*P* < 0.05 (vs dex group).

**Figure 7:** The main results and significance of this experiment.

## Data Availability

The data used to support the findings of this study are available from the corresponding author upon request.
